# Analysis of Proteomic Characteristics of Peripheral Blood in Preeclampsia and Study of Changes in Fetal Arterial Doppler Parameters Based on Magnetic Nanoparticles

**DOI:** 10.1155/2021/7145487

**Published:** 2021-11-02

**Authors:** Xundan Zhou, Lei Qu, Wenting Zhang, Fang Yang, Xiaoxia Hou, Shaoli Wang

**Affiliations:** ^1^Center of Ultrasound in Medicine, Northwest Women and Children's Hospital, Xi'an, China; ^2^Department of Clinical Laboratory, Northwest Women and Children's Hospital, Xi'an, China; ^3^Department of Obstetrics, Northwest Women and Children's Hospital, Xi'an, China

## Abstract

**Background:**

Traditional mass spectrometry detection methods have low detection efficiency for low-abundance proteins, thus limiting the application of proteomic analysis in the diagnosis of preeclampsia. Magnetic nanomaterials have good superparamagnetism and have obvious advantages in the field of biological separation and enrichment.

**Aim:**

The objective of this study is to explore the value of superparamagnetic iron oxide nanoparticles in the proteomic analysis of preeclampsia.

**Materials and Methods:**

42 patients and 40 normal pregnant women were selected in this study for analysis. Gene Ontology enrichment analysis and Kyoto Encyclopedia of Genes and Genomes (KEGG) enrichment analysis were performed to evaluate the function of these differential proteins. Proteomic analysis was used to analyze the differential proteins. Color Doppler ultrasound technology was used to detect changes in the blood flow of the fetal umbilical artery and cerebral artery.

**Results:**

16 differential proteins in the serum of pregnant women with preeclampsia and normal pregnant women were detected. The 16 proteins are mainly related to angiogenesis and endothelial function proteins, coagulation cascade proteins, placental growth factor, and so on. Biological function analysis revealed that these proteins are mainly enriched in the nuclear factor kB (NF-*κ*B) signaling pathway. Moreover, our data suggested that compared with the fetus in the uterus of normal pregnant women, the umbilical artery S/D, PI, and RI of the fetus in preeclampsia were greatly increased, and the cerebral artery S/D, PI, and RI were greatly decreased.

**Conclusion:**

Biological function analysis revealed that 16 proteins are mainly enriched in the NF-*κ*B signaling pathway. Compared with the normal group, the umbilical artery S/D, PI, and RI of the preeclampsia group were greatly increased, and the cerebral artery S/D, PI, and RI were all greatly reduced. Our findings provided a more comprehensive reference for us to study the mechanism of preeclampsia at the molecular level and also provide data support for the screening of relevant markers for early diagnosis of preeclampsia.

## 1. Introduction

Preeclampsia refers to a disease in which the blood pressure of a pregnant woman is normal before pregnancy, but symptoms such as high blood pressure and urine protein appear after 20 weeks of pregnancy. According to relevant epidemiological survey data, the worldwide incidence of preeclampsia is about 5%, which is one of the main causes of death of pregnant women [1]. In addition, more than 15% of preeclampsia worldwide are caused by preeclampsia [2]. As a systemic inflammatory disease, preeclampsia will not only damage the heart, liver, kidney, nerve, blood, and other organs and systems during pregnancy but also increase the risk of placental abruption, fetal intrauterine growth restriction, and HELLP syndrome [3, 4]. Current studies believe that the occurrence of preeclampsia is affected by the combined effects of various factors such as excessive oxidative stress, impaired angiogenesis, abnormal implantation of the placenta, and abnormal immune regulation [5, 6]. In-depth exploration of the pathogenesis of preeclampsia, looking for effective early predictive indicators, can provide guidance for early detection and timely treatment of preeclampsia.

As an important component of human cells and tissues, protein is the material basis for life and life activities. Since the implementation of the Human Genome Project, proteomics has become one of the core contents of life science research. Scholars conduct research on specific roles played by proteomics in different time and space. And use the functional mechanism of protein and its regulation of human immunity and metabolism to provide a theoretical basis for clinical disease diagnosis, new drug development, and metabolism research [7, 8]. Therefore, screening the protein in the blood of pregnant women with preeclampsia, and comparing them with normal pregnant women, finds out the different proteins, which is of great significance to the diagnosis and treatment of preeclampsia.

In human blood, quantitative detection of protein is often used for early diagnosis of diseases. However, since most of the proteins with regulatory effects are low-abundance proteins, it is difficult to enrich, separate, detect, and identify low-abundance proteins. Therefore, traditional mass spectrometry detection methods have low detection efficiency for low-abundance proteins, which limits the application of proteomic analysis in disease diagnosis. In recent years, due to the wide application of nanomaterials in medicine and biology, many scholars have noticed the advantages of nanomaterials in the field of biological separation: small size, high plasticity, and unique physical and chemical properties [9, 10]. With the deepening of research on the separation and enrichment of proteins/peptides, the application of functionalized nanomaterials in the enrichment and identification of low-abundance proteins has become a hot research direction. By combining the nanofluid enrichment device with resonance energy transfer technology for the detection of trace proteins, Wang et al. found that the detection limit of this method for bovine serum albumin was significantly lower than that of traditional detection methods [11]. Therefore, this study used functionalized magnetic iron oxide nanoparticles to enrich and identify the proteome in the peripheral blood of patients with preeclampsia, aiming to explore the proteomic characteristics of the peripheral blood of patients with preeclampsia.

A timely understanding of the developmental status of the fetus in pregnant women with preeclampsia can help to take corresponding measures to reduce the risk of fetal birth defects. Color Doppler Flow Imaging (CDFI) is a noninvasive and highly reproducible clinical diagnosis technology that can understand the development of the fetus in the uterus by collecting ultrasound images, blood flow, and other information [12]. The fetal umbilical artery is connected to the placenta and maternal arteries, and the function of the placenta and intrauterine growth of the fetus can be understood according to its blood flow information [13]. Cerebral arteries are one of the most important blood vessels in the fetal brain, and the blood flow of the cerebral arteries can directly reflect the development of the fetal brain [14]. Therefore, this study analyzed the changes in Doppler parameters of the umbilical and cerebral arteries of the fetus in pregnant women with preeclampsia and normal pregnant women and provided references for timely detection and correction of fetal dysplasia.

## 2. Materials and Methods

### 2.1. Research Object

42 preeclampsia patients admitted to our hospital from January 2020 to June 2020 were selected as the research objects. The inclusion criteria of the patients are as follows: (1) set up a file in our hospital for pregnancy health check and finally give birth in this hospital; (2) singleton pregnancy; (3) 18-35 years old, and the gestational age determined by ultrasound is more than 28 weeks; (4) complete clinical data and voluntary participation in this study; (5) meet the diagnostic criteria for preeclampsia. Patients who meet the following criteria will be excluded: (1) with pregnancy-induced hypertension, hyperglycemia, anemia, and other pregnancy complications; (2) artificial insemination. In addition, 40 normal pregnant women whose general data such as age, gestational age, and parity are comparable to those of preeclampsia patients were selected as the control group for the study.

### 2.2. Extraction of Protein and Enrichment of Protein by Magnetic Nanoparticles

The serum samples of preeclampsia and healthy pregnant women were mixed into 10 biological replicates. 0.5 mL of cell lysate was added to 20 mixed serum samples to be tested and centrifuged (15 min, 18000 × g) after sonication in an ice bath for 15 min. Aspirate the supernatant obtained by centrifugation, and use the diquinoline acid (BCA) method for protein quantification. After quantification, a 20 *μ*m sample was taken for protein enrichment. In order to improve the enrichment efficiency of low-abundance proteins, this study used magnetic iron oxide nanoparticles functionalized with amino groups for protein enrichment. The principle is to use the chemical bonding properties between disulfide bond-containing magnetic nanoparticles and aldehyde group-containing protein to specifically enrich the protein in the presence of a catalyst and finally use a reducing agent to break the bonded chemical bond to release the protein. The whole enrichment process can maintain the integrity of the protein, and the operation is simple, and at the same time, it is highly efficient and economical. The specific steps of enrichment are shown in Figure 1. First, add an appropriate amount of functionalized magnetic nanoparticles (the mass ratio of protein to iron oxide nanoparticles is 2 : 5) into the protein sample solution, use the superparamagnetism of the magnetic nanoparticles, and use a magnet to bond the protein-bound magnetic nanoparticles separate from the supernatant. The eluent is used to remove the nonchemically bonded proteins on the surface of the magnetic nanoparticles, complete the purification and enrichment of the proteins, and then use the released proteins for mass spectrometry analysis.

### 2.3. Collection of Separation and Enrichment Protein Data

First, perform Data-Dependent Acquisition (DDA): dissolve the enzymatically hydrolyzed peptide sample in 25 *μ*L of 0.1% formic acid aqueous solution (including iRT standard peptide), and then place 5 *μ*L of the sample in the EASY-Nano-LC chromatography system. The sample is transferred to the precolumn (transfer flow rate: 4.5 *μ*L/min), and then, the sample is analyzed (analysis flow rate: 300 nL/min). Mass spectrometry data was collected by the Orbitrap Fusion Lumos Tribrid mass spectrometer (Thermo Company, USA). Then, carry out Data-Independent Acquisition (DIA): each sample takes 2 *μ*g peptides for independent data mass spectrometry test, and the test time is 2 h. After the test, the separation is performed on the same chromatographic system as DDA, and the instrument for mass spectrometry data collection is the same as that of DDA.

### 2.4. Qualitative, Quantitative, and Biological Function Analysis of Protein

In this study, ProteinPilot and SWATH 2.0 proteomic analysis software were used to analyze the protein qualitatively and quantitatively. Use the OmicsBeam protein data analysis platform to perform Gene Ontology (GO) analysis on the selected differential proteins. Complete the pathway analysis of differential proteins through the Kyoto Encyclopedia of Genes and Genomes (KEGG) database, and clarify the main signal transduction pathways and metabolic pathways of differential proteins involved in life activities.

### 2.5. Collection of Fetal Artery Doppler Parameters

The Philips i U22 color Doppler ultrasound system produced by Philips in the Netherlands was used to perform ultrasound examinations on all subjects. During the examination, the pregnant woman took the supine position, rested quietly for about 5 minutes, and then started the ultrasound examination. First, perform routine second-order ultrasound scanning to detect fetal heart rate, body weight, abdominal circumference, and other conventional biological indicators, and evaluate the fetal growth in the uterus. Then, switch to the color mode to measure the Doppler parameters of the fetal umbilical artery and cerebral artery blood flow.

Umbilical artery Doppler parameter detection: set the probe frequency to 3.5 MHz, select the free-floating segment of the umbilical artery for Doppler sampling when the fetus is quiet, and collect the umbilical artery blood flow image and freeze it. Use the analysis software that comes with the instrument to analyze the peak systolic velocity (PSV) of the umbilical artery, end-diastolic blood flow velocity (EDV), pulsatility index (PI), and resistance index (RI), and calculate the ratio of PSV to EDV (S/D).

Cerebral artery Doppler parameter detection: after the second-order ultrasound clarifies the cross-section of the fetal brain, slowly move the probe until the fetal bilateral sphenoid wings can be observed, and switch the ultrasound to color mode to detect the fetal intracranial blood flow information. Sampling is taken at the branch of the cerebral artery and the carotid artery, and the image is frozen when the fetus is breathing smoothly. The analysis of related blood flow parameters is the same as the method used for umbilical artery collection.

### 2.6. Statistical Analysis

This study used SPSS v.23.0 and GraphPad Prism v.8.0 software for data analysis. Quantitative data are expressed in the form of mean ± standard deviation. Two-group comparisons, multigroup comparisons, and pairwise comparisons between multiple groups were performed by the *t*-test, analysis of variance, and SNA-Q test. In the protein difference analysis, the difference of protein abundance is more than 1.3 times as the difference protein. In the analysis of all data, *P* < 0.05 indicates that the difference is statistically different.

## 3. Results and Discussion

### 3.1. Magnetic Nanoparticle Identification

In order to confirm the protein enrichment effect of magnetic iron oxide nanoparticles, we determined the characterization and disulfide bond content of magnetic nanoparticles used in the study. It can be seen from the TEM image that the magnetic nanoparticles are uniform in size and have good dispersion (as shown in Figure 2(a)). By drawing the sulfhydryl standard curve, it can be seen that the absorbance of magnetic nanoparticles has a good fit (as shown in Figure 2(b)).

### 3.2. Proteomic Characteristics and GO Analysis

Based on the protein enrichment effect of magnetic iron oxide nanoparticles, we performed protein profile analysis on 20 serum samples. After analysis, 297 proteins with clear annotations were obtained. Among them, the main functions are classified into angiogenesis, coagulation cascade, complement and inflammation, endothelial function regulation, and immune regulation. By comparing the protein characteristics of serum samples of 10 preeclampsia and 10 normal pregnant women, we found 16 proteins with significant differences, and the multiples of difference were all higher than 1.3. Through cluster analysis, it is found that these differential proteins can clearly distinguish the serum samples of pregnant women with preeclampsia and normal pregnancy. GO analysis of differential proteins found that the biological process (BP) mainly involves blood coagulation, fibrin clot formation, positive regulation of growth, and positive regulation of epithelial cell proliferation (as shown in Figure 3). Cellular component (CC) is mainly enriched in blood microparticles, collagen-containing extracellular matrix, and vesicle lumen (as shown in Figure 4). Molecular function (MF) is mainly enriched in glycosaminoglycan binding, growth factor activity, and heparin binding (as shown in Figure 5). The coordination between different proteins is called the biological function of the protein. This study is based on the pathway online database to analyze the biological function of the differential protein. After analysis, it is found that the above-mentioned differential proteins are mainly enriched in the nuclear factor kB (NF-*κ*B) signaling pathway.

### 3.3. Changes of Fetal Umbilical Artery Blood Flow

By comparing the Doppler parameters of the umbilical artery of the fetus in the uterus of pregnant women, it was found that the S/D, PI, and RI of the umbilical artery of the fetus in preeclampsia were greatly higher than those in the normal pregnancy group (*P* < 0.05), as shown in Table 1 and Figure 6.

### 3.4. Changes in Fetal Cerebral Arterial Blood Flow

By comparing the Doppler parameters of the cerebral arteries of the fetus in the uterus of pregnant women, it was found that the S/D, PI, and RI of the middle cerebral artery of the fetus in preeclampsia were greatly lower than those in the normal pregnancy group (*P* < 0.05), as shown in Table 2 and Figure 7.

### 3.5. Discussion

With the deepening of proteomic research, analyzing the specific pathogenesis of preeclampsia through differential proteins has become a hot spot in clinical research. At present, clinical analysis of the proteomic characteristics of pregnant women with preeclampsia mainly focuses on the patient's blood, urine, amniotic fluid, cerebrospinal fluid, etc. Among them, blood has become the main fluid for protein analysis in preeclampsia due to its convenient collection and high detection accuracy. Sample [15]. However, the current mass spectrometry detection technology mainly includes three processes for protein enrichment, coupling, cleaning, and release, but it is easy to cause the loss of low-abundance proteins during cleaning, which affects the research results [16, 17]. Therefore, it is necessary to find new technical means to reduce the loss of low-abundance proteins during the cleaning process. As a new type of material, magnetic nanomaterials have many advantages such as high dispersibility, biocompatibility, and superparamagnetism and are widely used in the biochemical field [18–20]. Superparamagnetism refers to a ferromagnetic substance with a single domain structure when the particle is smaller than the critical size. It exhibits paramagnetic characteristics when the temperature is lower than the Curie temperature and higher than the transition temperature, but its paramagnetic susceptibility is much higher under the action of an external magnetic field. The magnetic susceptibility of general paramagnetic materials [21–23]. The superparamagnetism of nanomaterials makes it extremely easy to be separated, which increases the advantages of nanomaterials in the field of biological separation and enrichment.

Based on the enrichment of magnetic iron oxide nanoparticles, this study analyzed the proteomic characteristics of the peripheral blood of pregnant women with preeclampsia and pregnant women with normal pregnancy. It was found that 16 proteins in the serum of patients with preeclampsia were significantly increased compared with normal pregnant women. Among these 16 differential proteins, many proteins have been proved to be closely related to the development of endothelial vascular injury diseases (even preeclampsia). For example, angiotensin disorders can cause cardiovascular disease by raising blood pressure; elevated fibrinogen can aggravate the inflammatory response in pregnant women; placental growth factor can promote placental angiogenesis and has a nourishing effect on the growth of placental cells [24–26]. This provides a more comprehensive reference for us to study the mechanism of preeclampsia at the molecular level and also provides data support for the screening of relevant markers for early diagnosis of preeclampsia. Functional proteomics is an analysis method that provides specific biomarkers for diseases by identifying specific proteins and their related pathways. Through biological function analysis, this study found that the NF-*κ*B signaling pathway is greatly different in the serum of preeclampsia patients and normal pregnant women. As we all know, the NF-*κ*B pathway plays a key role in regulating the growth and repair of vascular endothelial cells. Zhao and other scholars indicated in the study that inhibiting the activity of the NF-*κ*B pathway can reduce the inflammatory response of endothelial cells [27]. Lin et al. also confirmed that by regulating the NF-*κ*B pathway, it can inhibit the inflammatory cascade and improve the endothelial damage induced by high glucose [28].

In order to minimize the risk of adverse pregnancy outcomes for pregnant women with preeclampsia, it is necessary to monitor the growth of the fetus in the uterus, so as to take effective measures to intervene in time. At present, common clinical methods to monitor the fetal development in utero include fetal electronic monitoring, amnoscopy, and pregnant women's self-calculated fetal movement. However, fetal electronic monitoring can only be monitored when the fetus has obvious hypoxia, and it is not sensitive to early fetal abnormalities. Although the amnoscopy has high sensitivity, it is an invasive operation and can easily cause infections of the mother and fetus. In addition, the amnoscopy is difficult and complicated to operate, which is not conducive to dynamic monitoring. The self-calculated fetal movement of pregnant women is too subjective, and the clinical guidance value is low. In recent years, CDFI has been used in the dynamic monitoring of intracranial injuries, heart disease, liver cancer, and other diseases due to its advantages of noninvasive, intuitive, safe, and dynamic monitoring [29–31]. And with the rapid development of CDFI, it has become a convenient method in obstetrics and gynecology examinations [32]. The umbilical cord is an important hub connecting the fetus and the mother, as well as the main tool for the transportation of fetal nutrition and metabolites. Therefore, the blood flow state of the umbilical artery is related to the growth and development of the fetus, and the intrauterine growth of the fetus can be understood by detecting the blood flow of the umbilical artery. In this study, CDFI technology was used to collect fetal umbilical artery blood flow. After comparison, it was found that the fetal umbilical artery S/D ratio and PI and RI of the preeclampsia group were greatly higher than those of the normal pregnancy group. These suggest that the fetal umbilical artery blood flow resistance in the preeclampsia group is increased, and the blood flow speed is reduced, which may increase the risk of neonatal distress, hypoxia, and anemia.

The middle cerebral artery is a branch of the internal carotid artery and the main blood vessel for the cerebral blood supply. Through the blood flow changes in the middle cerebral artery of the fetus, we can understand the blood circulation in the brain. In addition, the brain is most sensitive to the body's hypoxia or ischemia, which makes the detection of cerebral arterial blood flow an effective indicator for evaluating fetal intrauterine growth [33]. At the same time, the position of the fetal cerebral artery is less affected by the fetal position, movement, and respiration, and the error produced by the CDFI measurement is relatively small. Under normal circumstances, with the increase of maternal pregnancy time and the development of fetal cerebral blood vessels, the diameter of fetal cerebral arteries will increase and the blood flow resistance will decrease to achieve the purpose of increasing blood supply to the brain [34].

In this study, the changes of intrauterine fetal cerebral arterial blood flow parameters in pregnant women with preeclampsia were detected by CDFI, and it was found that the fetal S/D ratio and PI and RI of the preeclampsia group were greatly lower than those of the normal pregnancy group. This may be because the main pathological feature of preeclampsia is the damage of maternal vascular endothelial cells, which makes the blood perfusion of organs including the uterus placenta decrease. When the placental blood perfusion drops, it will increase the vascular resistance and affect the material exchange between the mother and the placenta. The reduced blood flow exchanged between the mother and the placenta will affect the blood oxygen supply of the fetus. When the fetus has anemia or hypoxia in the uterus, in order to ensure the normal blood supply to the fetus's brain, the blood resistance of the cerebral arteries will decrease and the flow rate will increase.

## 4. Conclusion

Biological function analysis revealed that 16 proteins are mainly enriched in the NF-*κ*B signaling pathway. Compared with the normal group, the umbilical artery S/D, PI, and RI of the preeclampsia group were greatly increased, and the cerebral artery S/D, PI, and RI were all greatly reduced. Our findings provided a more comprehensive reference for us to study the mechanism of preeclampsia at the molecular level and also provide data support for the screening of relevant markers for early diagnosis of preeclampsia.

## Figures and Tables

**Figure 1:** Enrichment process of magnetic iron oxide nanoparticles and protein.

**Figure 2:** Characterization of magnetic iron oxide nanoparticles: (a) transmission electron micrograph of magnetic nanoparticles; (b) the sulfhydryl standard curve of magnetic nanoparticles.

**Figure 3:** Gene Ontology (GO) analysis of biological processes.

**Figure 4:** GO analysis of cellular component.

**Figure 5:** GO analysis of molecular function (MF).

**Figure 6:** Changes of Doppler parameters of umbilical artery blood flow: (a) the ratio of umbilical artery peak systolic velocity to end-diastolic blood flow velocity (S/D); (b) umbilical artery pulsatility index; (c) umbilical artery blood flow resistance index.

**Figure 7:** Changes of Doppler parameters of middle cerebral blood flow: (a) the ratio of middle cerebral artery peak systolic velocity to end-diastolic blood flow velocity (S/D); (b) pulsatility index of middle cerebral artery; (c) blood flow resistance index of middle cerebral artery.

**Table 1:** Changes of Doppler parameters of umbilical artery blood flow.

Grouping	S/D	PI	RI
Preeclampsia	2.79 ± 0.31	1.25 ± 0.17	0.78 ± 0.09
Normal	2.16 ± 0.23	0.94 ± 0.12	0.62 ± 0.10
*t*	10.413	9.497	7.623
*P*	<0.001	<0.001	<0.001

**Table 2:** Changes of Doppler parameters of middle cerebral artery blood flow.

Grouping	S/D	PI	RI
Preeclampsia	4.13 ± 0.40	1.42 ± 0.16	0.68 ± 0.07
Normal	5.56 ± 0.58	1.79 ± 0.28	0.89 ± 0.11
*t*	13.051	7.391	10.362
*P*	<0.001	<0.001	<0.001

## Data Availability

All the raw data could be accessed by contacting the corresponding author if someone qualified need it.
